# Diagnostic Values of Advanced Glycation End Products and Homocysteine in Patients with Alzheimer's Disease and Sarcopenia

**DOI:** 10.1155/2022/8949048

**Published:** 2022-09-09

**Authors:** Xuelian Zhang, Yunxia Meng, Weiwei Zhang, Luhang Shi, Xia Liu, Lijuan Zhang, Qiaoling Liu

**Affiliations:** Geriatrics Department, The First People's Hospital of Lianyungang, Xuzhou Medical University Affiliated Hospital of Lianyungang, The First Affiliated Hospital of Kangda College of Nangjing Medical University, Jiangsu 222002, Jiangsu, China

## Abstract

This study is aimed at exploring the diagnostic value of advanced glycation end products (AGEs) and homocysteine (Hcy) in Alzheimer's disease (AD) complicated with sarcopenia (SP) and to analyze the risk factors related to AD complicated with SP. A total of 168 patients admitted to our hospital from November 2019 to December 2021 were enrolled. Patients were divided into the NC (no SP and AD) group with 29 cases, the AD group with 39 cases, the AD+SP group with 35 cases, and the SP group with 65 cases. The general information, Mini-Mental State Examination (MMSE) scores, and serum levels of AGEs and Hcy among the four groups were compared. Unordered logistic regression was used to analyze the influencing factors of SP patients complicated with dementia. The AGE level was higher in the AD or AD+SP group than the NC or SP group (*P* < 0.05). There was no significant difference between the SP group and the NC group or between the AD group and the AD+SP group (*P* > 0.05). The Hcy level was higher in the SP or AD group than the NC group (*P* < 0.05). There were no significant differences between the AD group and NC group or between the SP group and AD+SP group (*P* > 0.05). The ROC curve of serum AGEs and Hcy for the diagnosis of AD showed that the area under curve (AUC) was 0.887, *P* < 0.05 (95% CI: 0.821-0.954, sensitivity: 80.95%, specificity: 73.81%) and 0.7423, *P* < 0.05 (95% CI: 0.6382-0.8465, sensitivity: 60.42%, specificity: 57.59%), respectively. The ROC curve of serum AGEs and Hcy for the diagnosis of SP showed that the AUC was 0.5533, *P* > 0.05 (95% CI: 0.4294-0.6771) and 0.8744, *P* < 0.05 (95% CI: 0.8006-0.9483). Age (*P* < 0.001), depression (*P* = 0.001), malnutrition (*P* = 0.002), and BMI (*P* < 0.001) were independent influencing factors of SP complicated with AD in elderly inpatients. In conclusion, combined serum AGEs and Hcy had a good diagnostic value for AD combined with SP, which may be helpful for early detection of patient condition.

## 1. Introduction

Alzheimer's disease (AD), a common clinical degenerative disease of the central nervous system, is mainly characterized by destabilization of the neuronal network and neuronal death. Its two major pathological features are the formation of extracellular insoluble senile plaques and the tangles of intracellular neuronal fibers [1, 2]. The etiology and pathogenesis of senile dementia are still unclear, and it is mostly considered to be a complex brain disease involving multiple factors and multiple pathological pathways. Sarcopenia (SP) is a new type of geriatric syndrome that has become popular in recent years, which refers to an age-related decrease in muscle mass, accompanied by the decrease in muscle strength and/or physical function [3]. In China, SP is still in the stage of low awareness rate and lack of awareness of prevention and treatment. The main clinical manifestations of SP are the decrease in mobility and body balance and difficulty in completing daily activities such as walking and sitting, and adverse events, such as falls, fragility fractures, and osteoporosis, are prone to occur [4]. Age, exercise, diabetes, inflammatory cytokines, vitamin D, hormone levels, etc., are all high-risk factors for SP, but their correlations need further study.

Increasing studies have shown that AD and SP have many overlapping phenomena in the pathogenesis and pathological changes [5, 6]. Studies have reported that at least 40% of patients diagnosed with SP have pathological changes in AD [7]. Studies have shown that early intervention for SP makes the disease reversible to a certain extent [8], but the current treatment for AD only controls symptoms and delays the progression of the disease. Therefore, it is crucial to study the possible common pathogenesis of AD and SP and their relationship and thus to explore their common biomarkers, so as to implement early diagnosis and intervention for AD and SP patients.

In recent years, the relationship between advanced glycation end products (AGEs) and AD has attracted more and more attention. AGEs are stable end products generated by nonenzymatic reaction between free amino groups, such as groups of proteins, lipids, nucleic acids, and other macromolecules and carbonyl groups of glucose or other reducing sugars. Under normal conditions, AGEs-modified proteins act as a signal to participate in the removal of aging tissues and structural reconstruction in the body. Under pathological conditions, AGEs can cause the abnormity of cellular structure and function of tissues, resulting in a series of pathological changes [9]. Current research shows that AGEs accelerate human aging and are related to the occurrence of a variety of chronic degenerative diseases [10], and it is believed that AGEs may also be one of the causes of AD. However, there are few studies related to SP and AGEs, which needs further exploration.

Homocysteine (Hcy) belongs to a noncoded amino acid and a transitional product of methionine cycle. As a neurotoxin, Hcy maintains normal physiological level by remethylation to methionine, among which vitamin B6, folic acid, and B12 are common nutrients in the diet [11]. Recent studies have also demonstrated that Hcy is a risk factor for cardiovascular and cerebrovascular diseases [12]. Geisel et al. have shown that Hcy can activate N-methyl-D-aspartate receptor (NMDAR), leading to neuronal death in the hippocampus [13]. Hcy also has an excitotoxic effect on hippocampal neurons, inducing dementia [13]. Importantly, Hcy was considered a main risk coefficient for AD as high plasma concentrations were related to the progression of this disease [14]. High Hcy serum concentration was also associated with behavioral and psychological evidence of AD [15]. However, its relation to SP and whether it could be used as a biomarker for early diagnosis of SP remains unexplored.

Therefore, this study is aimed at explore the diagnostic values of AGEs and Hcy underlying the pathogenesis of AD and SP and possible relationship between them and search possible laboratory markers with diagnostic value, which provides clinical possibilities for early detection, diagnosis, and prevention of the disease.

## 2. Materials and Methods

### 2.1. General Data

A total of 168 patients admitted to the Department of Neurology in our hospital from November 2019 to December 2021 were collected, including 102 males and 66 females, with an age distribution of 64-88 years, and an average age of 71.40 ± 6.18 years. This study was approved by the Ethics Committee of our hospital, and the informed consent was signed before treatment. Inclusion criteria are as follows: (1) age ≥ 60 years old; (2) well informed and agreed to participate in this study; (3) able to read, write, and speak Chinese normally and able to complete the questionnaire; and (4) able to move freely and able to complete pace, grip strength, and balance tests. Exclusion criteria are as follows: (1) a history of intracranial infection and other serious autoimmune diseases; (2) serious diseases (malignant tumors, severe liver, and kidney damage), etc.; and (3) MRI or CT confirmed cerebral infarction or cerebral hemorrhage and hemiplegia patients. According to whether the patients had SP and dementia, they were divided into the no SP and AD (NC) group (*n* = 29), the AD group (*n* = 39), the AD and SP group (*n* = 35), and the SP group (*n* = 65).

### 2.2. Data Collection

Within 4 h after admission, nervous system physical examination of all the inclusive research objects was performed by professional neurologists with information and medical history recorded. The anticoagulation tubes were used to store the fasting elbow venous blood drawn early in the morning. After 1 h, the serum was separated by centrifugation of 3000 r/min for 10 min. The separated serum was dispensed with the frozen pipe to freeze up at -80°C refrigerator for detection of indicators such as blood biochemistry, serum AGES, and Hcy. Within 48 h of admission, the head CT or skull MR, cerebrovascular and carotid duplex ultrasound, electrocardiogram, chest X-ray, and other inspections were performed. Basic information, such as name, gender, age, height, and weight, were collected. Smoking, drinking, hypertension, diabetes history, and stroke history were collected. MMSE and HIS scale were evaluated. Body mass index = body weight/height^2^ (kg/m^2^). All experiments on humans were conducted in accordance with the Declaration of Helsinki (1964) and were approved by the ethical committee of the First People's Hospital of Lianyungang.

### 2.3. Detection of Serum AGEs and Hcy

Serum AGE and Hcy kits were purchased from Wuhan Canvest Biotechnology Co., Ltd. The frozen specimens (50 *μ*L of serum) were placed in a 37°C water bath for instant dissolution once obtained and then measured by double-sandwich enzyme-linked immunosorbent assay (ELISA). In the process, a full-wavelength GeminiXPS fluorescent microplate reader was used for analysis, and the experimental steps were shown in the instructions of the kit.

### 2.4. Analysis of Risk Factors

Diagnostic criteria for risk factors are as follows: (1) hypertension: had a history of hypertension or were taking antihypertensive drugs; systolic blood pressure ≥ 140 mmHg and/or diastolic blood pressure ≥ 90 mmHg measured in resting state for 2 consecutive times without taking antihypertensive drugs; (2) diabetes: had a history of diabetes or were taking hypoglycemic drugs/insulin to control blood glucose; fasting blood glucose (FBG) ≥ 7.00 mmol/L, 2 h postprandial glucose (2hPG) ≥ 11.10 mmol/L, with or without diabetes symptoms; (3) smoking: average smoking ≥ 10 cigarettes/day and duration >1 year; (4) drinking: drinking any beer, liquor, or wine, average ethanol intake ≥ 30 g/day and duration > 1 year.

### 2.5. Mini-Mental State Examination (MMSE)

The MMSE scale was currently the most commonly used and influential scale in the world. The scale included orientation, memory, calculation and attention, recall ability, and language ability. Language ability included naming ability, repetition ability, three-step commands, reading ability, writing ability, and structural ability, with a total score of 30 points, and it took about 5-10 minutes [16]. 27-30 points were normal, and <27 points were AD. Dementia criteria are as follows: illiteracy ≤ 17 points, primary school education (education years ≤ 6 years) ≤ 20 points, middle school (including technical secondary school) ≤ 22 points, and college and above (including junior college) ≤ 23 points. Dementia degree evaluation: 21-24 points were mild; 10-20 points were moderate; ≤9 points were severe.

### 2.6. Montreal Cognitive Assessment (MoCA)

Montreal Cognitive Assessment (MoCA) included visuospatial and executive function (0-5 points), attention (0-6 points), delayed recall memory (0-5 points), naming (0-3 points), language (0-3 points), abstraction (0-2 points), and orientation (0-6 points), with a total score of 30 points [17]. When the score was less than or equal to 18 points, the patient was identified as dementia. Dementia degree evaluation: 18-15 points were mild; 15-10 points were moderate; ≤9 points were severe.

### 2.7. Diagnosis of SP

This study used the diagnostic criteria of the Asian Working Group for Sarcopenia (AWGS) (2019) [3] to diagnose SP. (1) Appendicular skeletal muscle mass index (ASMI) measurement: it was measured by bioelectrical impedance analysis (Inbody S10), where ASMI < 7.0 kg/m^2^ for males and <5.7 kg/m^2^ for females were defined as the decline of skeletal muscle mass. (2) Grip strength measurement: it was measured by the grip strength tester (Xiangshan EH101). The research subjects were required to hold the grip strength meter with all their strength when standing, and the left and right hands were measured 3 times, respectively, and the maximum value was taken. Men < 28 kg and women < 18 kg were the decline of grip strength. (3) Physical activity ability: it was measured by the 6 m pace measurement method. The pace of ≤1.0 m/s was regarded as the decline of physical function. SP was diagnosed when a subject had a decrease in skeletal muscle mass accompanied by a decrease in grip strength or physical function.

### 2.8. Assessment of Mental State

The Geriatric Depression Scale (GDS-5) was used to evaluate the depressive symptoms of the research subjects. It contained 5 items totally, and the subjects answered “yes” or “no.” The answer “yes” was scored 1 point, “no” was scored 0 points, and the total score over 2 points indicated that there may be depressive symptoms [8].

### 2.9. Assessment of Nutritional Status

The nutritional status was assessed using the mini nutritional assessment-short form (MNA-SF), with 14 points as total scores, 12-14 points as normal nutritional status, 8-11 points as the risk of malnutrition, and 0 ~ 7 points to malnutrition [18].

### 2.10. Statistical Analysis

SPSS 20.0 software was used for statistical analysis of data. Measurement data were expressed as mean ± standard deviation, and ANOVA was used for comparison between groups; enumeration data was expressed as the number of cases (%), and chi-square test was used for comparison between groups; unordered logistic regression was used to analyze the influencing factors of SP patients complicated with AD. The area under the curve of AGEs and Hcy in the diagnosis of AD and SP; the corresponding sensitivity, specificity, and 95% confidence interval were calculated. The test standard was *α* = 0.05, and *P* < 0.05 was considered statistically significant.

## 3. Results

### 3.1. Comparison of Basic Data among Four Groups

Among the included patients, 65 (38.69%) were in the SP group, and 39 (23.21%) were in the AD group; 35 (20.83%) were in the AD+SP group, and 29 (17.27%) were in the NC group. Statistical analysis showed that there were significant differences in age, BMI, hypertension, DM, cerebrovascular disease, osteoporosis, education level, depression, and nutritional status among the patients in each group (*P* < 0.05 or *P* < 0.001). At the same time, there were no significant differences in gender, cardiovascular disease, currently smoking, falls in the last 12 months and daily medication > 4 kinds among the patients in each group (*P* > 0.05), as shown in Table 1.

### 3.2. Comparison of Serum AGE Level among Four Groups

There was a statistically significant difference in serum AGEs among four groups (*P* < 0.05.) Pairwise comparison showed that the level of AGEs in the AD group was higher than that in the SP group, and the difference was statistically significant (*P* < 0.05); the level of AGEs in the AD group was higher than that in the NC group, and the difference was statistically significant (*P* < 0.05); the level of AGEs in the AD+SP group was higher than that in the SP group, and the difference was statistically significant (*P* < 0.05); the level of AGEs in the AD+SP group was higher than that in the NC group, and the difference was statistically significant (*P* < 0.05); there was no significant difference between the SP group and the NC group or between the AD group and the AD+SP group (*P* > 0.05) (Figure 1).

### 3.3. Comparison of Serum Hcy Level among Four Groups

There was a statistically significant difference in Hcy among four groups. Pairwise comparison showed that the level of Hcy in the SP group was higher than that in the NC group, and the difference was statistically significant (*P* < 0.05); the level of Hcy in the AD group was higher than that in the NC group, and the difference was statistically significant (*P* < 0.05); the level of Hcy in the AD+SP group was higher than that in the NC group, and the difference was statistically significant (*P* < 0.05); there was no significant difference between the AD group and SP group or between the SP group and AD+SP group or between the AD group and AD+SP group (*P* > 0.05) (Figure 2).

### 3.4. Diagnostic Characteristic Curves of Subjects

The ROC curve of serum AGEs for the diagnosis of AD showed that the area under curve (AUC) was 0.887, *P* < 0.05 and 95% CI was 0.821-0.954, indicating that serum AGEs have a high diagnostic value for AD, and the critical value of serum AGEs for the diagnosis of AD was 518.5 ng/L, with a diagnostic sensitivity of 80.95% and a specificity of 73.81%. The ROC curve of serum AGEs for the diagnosis of SP showed that the AUC was 0.5533, *P* > 0.05 and 95% CI was 0.4294-0.6771, indicating that serum AGEs have no diagnostic value for SP (Figure 3).

The ROC curve of serum Hcy for the diagnosis of AD showed that the AUC was 0.7423, *P* < 0.05 and 95% CI was 0.6382-0.8465, *P* < 0.05, indicating that serum Hcy has a diagnostic value for AD, with a diagnostic sensitivity of 60.42% and a specificity of 57.59%. The ROC curve of serum Hcy for the diagnosis of SP showed that the AUC was 0.8744, *P* < 0.05 and 95% CI was 0.8006-0.9483, indicating that serum Hcy has a good diagnostic value for SP, and the critical value of serum Hcy for the diagnosis of SP was 34.5, with a diagnostic sensitivity of 88.10% and a specificity of 72.16% (Figure 4).

The ROC curve of combined AGEs and Hcy for the diagnosis of AD and SP showed that the AUC was 0.9311, *P* < 0.05; 95% CI was 0.8845-0.9818, *P* < 0.05; the sensitivity was 88.10%, and the specificity was 78.57%, indicating that combined serum AGEs and Hcy have a good diagnostic value for AD and SP (Figure 5).

### 3.5. Logistic Regression Analysis of the Influencing Factors of SP Complicated with AD in Elderly Inpatients

Taking the NC group as the reference group, the abovementioned statistically significant factors were incorporated into the disordered logistic regression model. The results showed that age (*P* < 0.001), depression (*P* = 0.001), malnutrition (*P* = 0.002), and BMI (*P* < 0.001) were all independent influencing factors in the SP+AD group, as shown in Table 2.

## 4. Discussion

AD, a neurological disease with a high incidence rate among middle-aged and elderly people, seriously affects the quality of life and physical and mental health of the elderly and also brings a heavy burden to the family and society. SP, an age-related decline in skeletal muscle mass, muscle strength, and/or physical activity, is associated with adverse outcomes in older adults, such as decreased functional status, falls, poor quality of life, and increased mortality [6]. SP is considered an important public health problem due to its important clinical, economic, and social consequences and has now been formally recognized as a muscle disease. More and more studies have shown that AD and SP have a common pathogenesis. Researches on the possible risk factors of AD and SP, early intervention, and early diagnosis are essential to improve the treatments of patients and reduce the burden on families and society.

There are many studies on the relationship between AGEs and AD, and the main mechanisms leading to the pathogenesis may be as follows: AGEs can lead to the occurrence and development of AD through a variety of ways, such as modifying A*β* and Tau proteins, triggering inflammatory responses, causing mitochondrial dysfunction, producing oxidative stress damage and affecting cell metabolism, the cycle of neurons, autophagy, and the permeability of the blood-brain barrier, etc. [19]. There are few studies on AGEs and SP, most of which show that AGEs play an important role in the regulation of calcium and phosphorus, increasing serum calcium ion concentration and improving neuromuscular activity, and can also bind to vitamin D receptors, increasing the production of osteocalcin and osteopontin [20]. A study has revealed that the reduced vitamin D level can affect the homeostasis of insulin resistance in the elderly, thereby promoting the occurrence of SP [21]. In this study, AGEs in the AD group and the AD+SP group were significantly higher than those in the NC group and the SP group, and the difference was statistically significant, which was consistent with literature reports, suggesting that AGEs may promote the occurrence and development of AD through the abovementioned various mechanisms. The sensitivity and specificity of AGEs for the diagnosis of AD were calculated by drawing the ROC curve. The ROC curve of serum AGEs for the diagnosis of AD showed that the AUC was 0.887, *P* < 0.05 and 95% CI was 0.821-0.954, indicating that serum AGEs had a high diagnostic value for AD, and the critical value of serum AGEs for the diagnosis of AD was 518.5 ng/L, with a diagnostic sensitivity of 80.95% and a specificity of 73.81%. The ROC curve of serum AGEs for the diagnosis of SP showed that the AUC was 0.5533, *P* > 0.05, and 95% CI was 0.4294-0.6771, indicating that serum AGEs had no diagnostic value for SP.

Hcy, a sulfur-containing amino acid, is involved in the methionine cycle and is the product of methionine demethylation [22]. Some cross-sectional studies and prospective longitudinal epidemiological studies have shown that high Hcy level may increase the risk of AD [23]. However, a recent study has demonstrated that the elevated Hcy level is not associated with the occurrence, severity and progression of AD [24]. Studies have shown that high Hcy level may have an independent role in the pathogenesis of SP, and some cross-sectional studies have also shown that Hcy level is upregulated in SP patients [25]. The KIM study has revealed that high Hcy level is associated with brain atrophy, but whether reducing Hcy level can delay the progression of dementia or prevent the progression of neurodegenerative disease requires further research [26]. The ROC curve of serum Hcy for the diagnosis of AD showed that the AUC was 0.7423, *P* < 0.05, and 95% CI was 0.6382-0.8465, *P* < 0.05, indicating that serum Hcy had a significant diagnostic value for AD, with a diagnostic sensitivity of 60.42% and a specificity of 57.59%. The ROC curve of serum Hcy for the diagnosis of SP showed that the AUC was 0.8744, *P* < 0.05, and 95% CI was 0.8006-0.9483, indicating that serum Hcy had a good diagnostic value for SP, and the critical value of serum Hcy for the diagnosis of SP was 34.5, corresponding to a diagnostic sensitivity of 88.10% and a specificity of 72.16%. The ROC curve of combined AGEs and Hcy for the diagnosis of AD and SP showed that the AUC was 0.9311, *P* < 0.05; 95% CI was 0.8845-0.9818, *P* < 0.05; the sensitivity was 88.10%, and the specificity was 78.57%, indicating that combined serum AGEs and Hcy had a good diagnostic value for AD and SP.

The results of this study showed that the risk of SP complicated with AD increased by 1.221 times per year as the elderly patients aged. Under normal circumstances, the muscle mass and muscle strength of the human body will change with age. For most people over 50 years old, the muscle mass of the legs will decrease at a rate of 1% to 2% per year, and the muscle strength will also decrease by 1.5% to 5.0% per year [27]. At present, the biggest known risk factor for AD is increasing age, as is proved in its prevalence. Therefore, in clinical work, attention should be paid to screening for SP and AD in elderly patients.

This study also showed that elderly inpatients with or at risk of malnutrition are more likely to develop SP complicated with AD compared with elderly inpatients with normal nutrition (OR = 4.907, 95% CI: 1.685-14.108, *P* = 0.002). This may be due to the fact that malnutrition can lead to lower serum albumin level in patients. Protein is a component of muscle, and low protein intake can lead to low muscle mass, which leads to SP. Studies have found that AD patients have a higher risk of malnutrition compared with people with normal cognitive function [28]. It can be seen that attention should be paid to the nutritional status of elderly inpatients clinically. For patients at risk of malnutrition, further screening for SP and AD should be performed, and interventions such as nutritional supplementation and exercise training should be taken as soon as possible.

It is worth noting that the risk of SP complicated with AD in the elderly patients with depression in this study was 10.873 times that of the elderly patients without depression. There may be common pathophysiological mechanisms between SP and mental disorders (depression, AD). Skeletal muscle can release neurotrophic factors that nourish neuron growth and differentiation during contraction, which can have a positive effect in mood changes [29]. In addition, depression can reduce appetite, and result in insufficient protein intake, thereby causing the decreased muscle mass. A meta-analysis by Taiwanese scholars also has shown that with exclusion of confounding factors such as age, gender, cognitive function, and physical activity; SP is positively correlated with depression (OR = 1.821, 95% CI: 1.160-2.859) [30]. There is also a significant correlation between depression and AD in the elderly. Neurodegenerative changes [26], vascular damage, and neuroinflammatory changes [31], etc., are the common pathophysiological mechanisms between depression and AD. Another meta-analysis has shown that the prevalence rate of depression in mild AD patients was 32% (95% CI: 27%-37%), that is, 1 out of every 3 mild AD patients has a simultaneous suffer from depression [32]. In conclusion, screening for depressive symptoms in the elderly is critical for identifying SP and AD.

## 5. Conclusion

The combined serum AGEs and Hcy have a good diagnostic value for AD complicated with SP, which can help to detect the patient's condition early. In addition, age, depression, malnutrition and BMI are independent influencing factors of SP complicated with AD in elderly inpatients. These patients should be given sufficient attention in treatment and daily life.

## Figures and Tables

**Figure 1:** Serum AGEs level in four groups. Note: ^∗^*P* < 0.05, vs. the NC group; ^#^*P* < 0.05, vs. the SP group.

**Figure 2:** Serum Hcy level in four groups. Note: ^∗^*P* < 0.05, vs. the NC group.

**Figure 3:** ROC curve of AGEs for the diagnosis of AD and SP.

**Figure 4:** ROC curve of serum Hcy for the diagnosis of AD and SP.

**Figure 5:** ROC curve of combined AGEs and Hcy for the diagnosis of AD and SP.

**Table 1:** Basic data in four groups.

Item	NC	SP	AD	AD+SP	*P*
Age (year)	80.59 ± 7.36	84.22 ± 7.13	87.88 ± 6.72	90.48 ± 5.21	<0.001
Gender					
Male	19 (65.52)	40 (61.52)	23 (58.97)	20 (57.14)	0.763
Female	10 (34.48)	25 (38.45)	16 (41.03)	15 (42.86)	
BMI (*x* ± *s*)	24.33 ± 2.58	21.62 ± 2.36	26.08 ± 3.11	21.64 ± 3.18	<0.001
Comorbidity					
Hypertension	21 (72.41)	36 (55.37)	34 (69.23)	27 (77.14)	0.008
DM	15 (51.72)	24 (36.91)	35 (89.74)	14 (40.00)	0.012
Cardiovascular disease	9 (31.03)	21 (32. 30)	16 (41.03)	15 (42.86)	0.071
Cerebrovascular disease	19 (65.52)	38 (58.44)	24 (61.54)	29 (82.85)	0.032
Osteoporosis	7 (24.08)	31 (47.68)	9 (23.08)	11 (31.43)	<0.001
Education level					
≤6 years	1 (3.44)	4 (6.15)	6 (15.38)	2 (5.71)	<0.001
>6 years and <12 years	14 (48.16)	28 (43.06)	20 (51.28)	26 (74.29)	
≥12 years	13 (44.72)	33 (50.75)	12 (30.77)	8 (22.86)	
Currently smoking	3 (10.32)	3 (4.61)	3 (7.69)	2 (5.71)	0.407
Falls in the last 12 months	8 (27.52)	2 (33.83)	12 (30.77)	9 (25.71)	0.476
Daily medication > 4 kinds	17 (58.48)	34 (52.29)	26 (66.66)	22 (62.85)	0.243
Depression	1 (3.44)	9 (13.84)	7 (17.95)	7 (20.00)	<0.001
Malnutrition	2 (6.88)	18 (27.68)	8 (20.51)	21 (60.00)	<0.001

**Table 2:** The influencing factors of SP and/or AD in each group.

Groups	Variables	*P*	SE	Wald *X*^2^	*P*	OR (95% CI)
SP	Intercept	3.784	1.856	4.387	0.035	—
	Age	0.046	0.023	8.201	0.004	1.028 (1.017-1.093)
	BMI	-0.392	0.059	44.384	<0.001	0.703 (0.619-0.770)
	Depression	2.108	0.676	9.703	0.002	7.764 (2.140-28.525)
	Osteoporosis	1.092	0.311	12.632	<0.001	2.897 (1.633-5.437)
AD	Intercept	-9.337	2.876	11.517	0.001	—
	Age	0.112	0.034	12.341	<0.001	1.112 (1.045-1.170)
	Education level ≥ 6 years	2.273	0.663	12.444	<0.001	10.144 (2.802-36.662)
	Malnutrition	1.056	0.532	4.521	0.032	2.954 (1.088-8.091)
	Depression	1.907	0.709	7.317	0.006	6.546 (1.675-25.524)
AD+SP	Intercept	-12.976	4.573	8.309	0.003	—
	Age	0.223	0.046	19.972	< 0.001	1.227 (1.138-1.392)
	BMI	-0.415	0.081	25.535	< 0.001	0.633 (0.549-0.768)
	Malnutrition	1.626	0.572	8.556	0.002	4.907 (1.685-14.108)
	Depression	2.419	0.810	9.338	0.001	10.873 (2.345-49.885)

The first *P* represented the regression coefficient. The second *P* is a parameter used to determine the result of a hypothesis test, with *P* < 0.05 indicates significance.

## Data Availability

The datasets used and/or analyzed during the current study are available from the corresponding author upon request.
